# Research on Video Target Detection and Tracking in Football Matches

**DOI:** 10.1155/2022/6951532

**Published:** 2022-07-31

**Authors:** Xiaoju Zou, Yuanling Huang, Nairun Zhou, Zuoming Fang

**Affiliations:** ^1^Department of Physical Education, Guangzhou City University of Technology, Guangzhou 510800, Guangdong, China; ^2^College of Physical Education, Guangdong University of Education, Guangzhou 510800, Guangdong, China

## Abstract

Computer vision is an interesting branch of artificial intelligence which is dedicated to how electronic devices can achieve the level of capabilities to perceive things just like ordinary human beings do. In order to solve the poor effect of video for the detection of target in football matches and the low accuracy of target tracking, this paper aims to make a deep exploration of the methods of video for the detection of target and tracking in football matches. The video moving for the detection of target method based on background model is used to extract the image in the background of the matching video which improves the light flow field. Secondly, the video differential image is acquired according to the difference of colors, the ghost target of the image in the video background model is scientifically determined, the ghost degree of the pixel points of the image is scientifically determined, and the flicker matrix of the target image is constructed. The number of pixels of the moving target is derived. A meanshift-based video target tracking algorithm is used in conjunction for the detection of target result to determine whether to track the target image until the overall video target tracking task is completed, move the central position of the target frame and background frame to the target position, select the best one to adapt to the target change, and determine whether to track the target image until the overall video target tracking task is completed. The simulation results suggest that the approach described in this study is capable of detecting and tracking moving objects, as well as improving target recognition and tracking accuracy.

## 1. Introduction

Computer vision is an interesting branch of the artificial intelligence which is dedicated to how electronic devices can achieve the level of capabilities to perceive things just like ordinary human beings do. Usually for implementation of this, electronic devices must be equipped with additional sensors which has the capability to enable these devices to view things just like an eye of the human being does. In addition, it is an interested research domain, because if these devices, both computers and robots, can achieve this capability, then it would be easier to perform various tasks which are reserved for human beings only. In addition, as per our understanding, AI based devices and systems are utilized to automate various activities, however, this is subjected to the feasibility of these activities in the problem domain. Moreover, in certain scenarios, these systems, i.e., AI based smart systems, are utilized for the regular assistance of the field experts in various domains of life such as in medical sector, a decision support system could help a doctor in the diagnosis process of the disease. For this purpose, computer vision uses cameras and computers to acquire and process visual information. The purpose of computer is to achieve people's understanding of vision. Computer vision is the intersection and combination of disciplines, including mathematics and image processing, as well as computer science. Video for the detection of target and tracking is a hot topic in the field of computer vision and has received much attention at home and abroad. Video for the detection of target and tracking is a process of inferring the position of moving target in video by computer. The main task is to accurately locate the target in each frame of the video, and then generate the motion track of the target, giving the complete area of the moving target in video at any time.

Sports videos are a highly frequent form of video in entertainment videos in everyday life, occupying a substantial share of daily entertainment life, and football-related videos in sports videos are extensively watched by sports video viewers. Football coaches may use the video to study the detailed data of the necessary movement, and players can use the video to record the associated data of their own movement, which can be retrieved from the target movement's track in the football match film. These requirements can be satisfied and met with the use of high-cost labour and material resources for football matches. As a result, this study investigates football video target recognition and tracking systems in depth.

The following are the paper's innovations: (1) detecting the video target of a competition using a background model and visual detection technology, then integrating for the detection of target findings with the basic meanshift video target tracking algorithm to track the identified target. (2) When compared to traditional teaching methods, the Intelligent Teaching System for Chinese as a foreign language proposed in this paper has a high level of overall stability and can significantly improve students' learning efficiency and teaching quality.

The remainder of the paper is divided into the sections listed below. A detailed review of the existing methodologies is reported in the section two of the paper where feasibility of every scheme along with expected issues are described. In section three, computer vision-based football video for the detection of target method based on the background model is reported where how the vision capability of the devices can be used. Meanshift-enabled target tracking algorithm is described in detail and how it is effective in resolving the scenarios. Results of the experimental observations were described in section five of the paper which is followed by the summary of the whole manuscript.

## 2. Related Work

In football video, the detection of target and tracking is of great importance to the analysis of football video, so it has received wide attention and obtained corresponding research results. Gao [1], aiming at the problems for the detection of target in football video, adopts the method of football video for the detection of target and tracking based on improved Gauss model. First, it deeply analyses the drawbacks of the model itself, converts color image to gray image, and dynamically expands in areas with small differences in video similarity, so as to improve the efficiency and accuracy for the detection of target and tracking in football video with Gauss model. The experimental results show that this method has a strong ability to deal with video interference in football matches and a large detection range, but it has the problem of low accuracy of detection [1]. Tian [2] puts forward a robust algorithm for football video for the detection of target and tracking in order to achieve the stable detection and tracking of football video targets. The image of the match video is matched and calibrated, and the moving target in the video is detected by the image cumulative difference map. To achieve efficiency for the detection of target, the matching complexity of video feature points is reduced through the corresponding strategies of network sampling, thus solving the problem of nonuniform concentration of image feature points in video. Intensity filter algorithm is used to improve the significance of the target in the match video, to filter out the unwanted false targets, to propose a scale calculation and area detection method based on the detected targets, and then to use Kalman filter to track the detected targets. The experimental results show that this method can detect the moving target accurately in football video, but it does not track the target steadily [2]. Zhou et al. [3] proposed a color space-based detection and tracking method which is robust to light due to the problem of target loss during the staggered motion of football video targets. Edge detection is performed on the relatively accurate moving target's binary image after converting the moving target's binary image extracted from the color space, using brightness detection to judge whether the filtered binary image is morphologically operated, and then converting the moving target's binary image extracted from the color space. After obtaining the minimal enclosing rectangle frame, the associated motion tracks of different color targets are produced, and the multi-target tracking of the football match video is accomplished. It can address the problem of video tracking target staggered motion loss target better than previous methods, but it has poorer detection accuracy [3]. Zou et al. [4] is widely used in many fields such as video surveillance and artificial intelligence for target tracking. In order to detect and track the moving target of football video quickly, a for the detection of target and tracking method combining Kalman filter and particle filter is proposed. Under the framework of Kalman filter, combined with particle filter to predict the location of moving objects, the method proposed in this paper is compared with a single Kalman filter method. The experimental results show that the proposed method has higher accuracy and better real-time performance, but due to the complexity of the process, the tracking effect is poor [4].

## 3. Football Video for the Detection of Target Method Based on Background Model

Computer vision is among the potential candidate solutions for the problems in hand. It is used to enable a system to perceive various things in a professional manner which preserve expected levels of the precision and accuracy.

### 3.1. Background Extraction of Optical Flow Field

Figure 1 shows the video for the detection of target process for a football match. Figure 1 shows that the image optical flow field in football match video mainly refers to the change of image brightness mode position in adjacent frames. The function of video target time is defined as (*x*(*t*), *y*(*t*)). The corresponding gray level of image point in video is *E*(*x*(*t*), *y*(*t*), *t*). Based on the video brightness and smoothing constraints, the formula (1) and formula (2) error functions are expressed as follows:

(1) $$\begin{array}{c} \varepsilon_{b}=E_{x}u+E_{y}u+E_{t}, \end{array}$$

(2) $$\begin{array}{c} \varepsilon_{c}=\sqrt{{\left(\bar{u}+u\right)}^{2}+{\left(\bar{v}+v\right)}^{2}};\varepsilon^{2}=\alpha^{2}\varepsilon_{c}^{2}+\varepsilon_{b}^{2}. \end{array}$$

In formulas (1) and (2), *ε*_*b*_ is the error set according to the constant video brightness constraint, *ε*_*c*_ is the error set according to the video smoothing constraint, $\bar{u}$ is the average value of *u* in the neighborhood of the video image, $\bar{v}$ is the average value of *v* in the neighborhood of the video image, *ε* is the total error, *α* is the measurement error constant, *E*_*x*_ is the gray corresponding to the midpoint of the game video (*x*, *y*), and *E*_*y*_ is the gray corresponding to the midpoint of the game video (*x*, *y*). The grayscale of the match video does not change when *E*_*t*_ is *t* [5, 6].

The markers of the moving target in the video must be obtained using the division of the optical flow field threshold, the markers must be taken as the center, and all points within the radius of the circle as the center should be taken as the target area points of the game video using the extended theory of the circle area. It is assumed that (*x*_*i*_(*i*), *y*_*i*_(*i*)) is the first marker point in the T-frame of the game video. The specific extent *D*_*t*_(*i*) to be covered by (*x*_*i*_(*i*), *y*_*i*_(*i*)) as the center of the circle is expressed by the following formula:

(3) $$\begin{array}{c} D_{t}\left(i\right)=\left\{\left(x,y\right)|\sqrt{{\left(x-x_{t}\left(i\right)\right)}^{2}+{\left(y-y_{t}\left(i\right)\right)}^{2}}\leq r\right\}. \end{array}$$

In formula (3), both *x* and *y* represent the target mark points in the football game video. The reasonable selection of radius *r* can ensure the coverage of all target areas and effectively reduce the background points of the target area in the video. The estimated *D*_*t*_ of the football game video target area in frame *t* in the game video is expressed by the following formula:

(4) $$\begin{array}{c} D_{t}=\overset{M_{t}}{\underset{i=1}{\cup }}D_{t}\left(i\right). \end{array}$$

In formula (4), *M*_*t*_ is the number of mark points in the *t* frame of the competition video. After obtaining the area *D*_*t*_ of the moving target in each frame of the video, the background corresponding to the image in the video is estimated according to the gray value of the points outside the target area. Assuming that *F*_*t*_(*x*, *y*) is a function for determining whether each point in frame *t* in the game video is the target area, according to the solution of obtaining the optical flow field of frame *N*, the fixed background area *USB* of the target area in the video image is eliminated. When the area of the image background in the football game video is extracted, the background model of the football game video target image is calculated by formula (5), expressed as

(5) $$\begin{array}{c} CB\left(x,y\right)=\frac{\sum_{t=1}^{N}f_{t}\left(x,y\right)\left(1-F_{t}\left(x,y\right)\right)}{\sum_{t=1}^{N}\left(1-F_{t}\left(x,y\right)\right)}. \end{array}$$

In formula (5), *N* is the number of frames of the input football game video image, and *f*_*t*_(*x*, *y*) is the gray value of the *t* frame image in the video at the (*x*, *y*) coordinate. After obtaining the fixed background area and background model of the video image, a frame image *I*, if it belongs to the pixel of the image background area, the difference between the background model of the football game video image and the image *I* is calculated and expressed as

(6) $$\begin{array}{c} I-CB=\underset{\left(x,y\right)\in UCB}{\cup }\left|I\left(x,y\right)-CB\left(x,y\right)\right|. \end{array}$$

In formula (6), *I*(*x*, *y*) is all pixels in image *I*. If the difference of the sum is greater than the set threshold, it indicates that the background of the game video changes greatly and the convective light field needs to be extracted again [7, 8]. The model of the video image color difference is expressed as

(7) $$\begin{array}{c} I_{D}\left(x,y\right)=\text{max}\left\{\left|R_{b}\left(x,y\right)-R_{k}\left(x,y\right)\right|,\left|G_{b}\left(x,y\right)-G_{k}\left(x,y\right)\right|,\left|B_{b}\left(x,y\right)-B_{k}\left(x,y\right)\right|\right\}. \end{array}$$

In formula (7), *R*_*b*_(*x*, *y*) is the color background image's value of pixel *R* in the football game video, *G*_*b*_(*x*, *y*) is the color background image's value of pixel *G* in the football game video, *B*_*b*_(*x*, *y*) is the color background image's value of pixel *B* in the football game video, *B*_*k*_(*x*, *y*)*G*_*k*_(*x*, *y*) and *B*_*k*_(*x*, *y*) are the three primary color values of the current frame image of the football game video, and the difference image formation can improve the integrity for the detection of target area of the football game video by using color information [9, 10].

### 3.2. Ghost Elimination of Video Target in Football Match

In the process of detecting the moving target of the game video, the pixel *x* of any image has a corresponding counter *f*_count_(*x*). If the moving target image pixel waiting to be detected is a foreground pixel, it is necessary to judge whether the image pixel in the background model is restrictive. If it has significant characteristics, the pixel *f*_count_(*x*) of the video frame waiting to be detected needs to be increased by 1, which is expressed as

(8) $$\begin{array}{c} f_{\text{count}}\left(x\right)=\left\{\begin{array}{cc} f_{\text{count}}\left(x\right), & f\left(x\right)=1\cap S\left(x\right)=1,\\ 0, & \text{else}. \end{array}\right. \end{array}$$

In formula (8), *f*(*x*) is the function of judging whether the image pixel *x* is a foreground image, *S*(*x*) represents the detection result of the significance of the background model saved in the detection target image relative to the pixel *x*, and the fuzzy set theory is introduced when the background of the football game video image is updated. *Z* represents the element set of the game video image, *z* is a certain kind of element *Z*={*z*}, and the fuzzy set *A* in *Z* is represented by the membership function *μ*_*A*_(*z*), The fuzzy set of football game video is an ordered pair composed of *z* value and corresponding membership function.

(9) $$\begin{array}{c} A=\left\{z,\mu_{A}\left(z\right)|z\in Z\right\}. \end{array}$$

In formula (9), *μ*_*A*_(*z*) describes the ghost degree of image pixels in the background model, and *z* describes the image pixels to be detected in the video image. When the pixel *f*_num_(*x*) of the video image is determined to be a ghost pixel, the corresponding image pixel needs to add *N*_0_ expansion operation. When the video pixel is determined not to be a ghost pixel during detection, *f*_num_(*x*) needs to subtract *N*_1_ expansion operation, which is expressed as

(10) $$\begin{array}{c} f_{\text{num}}\left(x\right)=\left\{\begin{array}{c} f_{\text{num}}\left(x\right)+N_{0},\;g\left(x\right)=1,\\ f_{\text{num}}\left(x\right)-N_{1},\;g\left(x\right)=0. \end{array}\right. \end{array}$$

In formula (10), *g*(*x*) represents whether the football game video pixel *x* is a function of ghost pixel determination, *N*_0_ and *N*_1_ represent fixed constants, and the range of *f*_num_(*x*) value is set in the interval [0, *φ*], *φ* represents the factor of time sampling. For this reason, the factor of secondary time sampling is expressed as

(11) $$\begin{array}{c} \phi =\varphi^{*}F\left(x\right). \end{array}$$

In formula (11), *F*(*x*) is a fuzzy function. By constructing the flicker matrix of the target pixel as the judgment principle, the degree of high-frequency disturbance of the video background is graded, and the matching threshold is set to *R*′, which is expressed as

(12) $$\begin{array}{c} R^{\prime }=\left\{\begin{array}{c} R\left(1+\lambda_{inc}\right),\;m\geq R_{b},\\ R\left(1-\lambda_{dec}\right),\;m≺R_{b}. \end{array}\right. \end{array}$$

In formula (12), *m* represents the data of the flicker matrix pixel of the target pixel of the football game video, and *R*_*b*_ represents the adaptive update boundary threshold of *R*′, and *λ*_*inc*_ and *λ*_*dec*_ represents the given parameters [11, 12].

## 4. Soccer Game Video Target Tracking Algorithm Based on Meanshift

Meanshift, frequently known as a mode-seeking methodology, is a nonparametric feature-space technique, i.e., it is used for the analysis of mathematics, for defining the maxima of a density function. Cluster analysis in computer vision and image processing are examples of application fields. Combined with the above football game video for the detection of target results based on the background model, set the space *R*^*d*^, *d* represents the dimension of the game video space, select *n* video sampling points *x*_*i*_, *i*=1,2,…, *n* in this space, and the basic form of meanshift vector at the reference video point *x* is expressed as

(13) $$\begin{array}{c} M_{h}\left(x\right)=\frac{1}{k}\sum_{x_{i}\in s_{h}}\left(x_{i}-x\right). \end{array}$$

In formula (13), (*x*_*i*_ − *x*) represents the offset of the game video target sample point *x*_*i*_ from the target reference point *x*, and *M*_*h*_(*x*) is the basic vector of meanshift algorithm [13, 14]. The sample point *x*_*i*_ in the target area of the game video is obtained in the density function *f*(*x*). When the density gradient value is greater than 0 or less than 0, the direction of the function gradient and the direction of density promotion are the same, and the direction of the sample sampled by the target in the *s*_*h*_ area is consistent with the direction of the density gradient. Therefore, the direction of the vector *M*_*h*_(*x*) of the meanshift algorithm is the same as the direction of the density gradient [15, 16].

Figure 2 shows the schematic diagram of mean value and Figure 3 shows the schematic diagram of mean value offset. In Figures 2 and 3, the square area is *s*_*h*_, and the direction pointed by the arrow is the vector to determine the offset of the target reference point *x*. The hollow circle represents *n* target sampling points in the foot video, which is satisfied with *x*_*i*_ ∈ *s*_*h*_, and the solid circle represents the reference point *x* of the vector target of the meanshift algorithm. The result of the basic vector *M*_*h*_(*x*) is offset to the maximum direction of the probability density of the sampling point of the moving target.

It can be seen from formula (13) that no matter how far the given target reference point *x* is from the target sampling point *x*_*i*_ in the football game video image area *s*_*h*_(*x*), the calculation result of the vector *M*_*h*_(*x*) of meanshift has the same impact. Therefore, the convergence speed of the video target reference point will become slow [17, 18]. In most cases, the closer the video target sampling point is to the target reference point, the greater the impact on the vector result will be. Therefore, different values will be given to the target sampling points with different distances from the moving target reference point. Formula (14) is the expansion formula of meanshift algorithm vector *M*_*h*_(*x*), which is expressed as

(14) $$\begin{array}{c} M_{h}\left(x\right)=\frac{\sum_{i=1}^{n}G\left(x_{i}-x/h\right)w\left(x_{i}\right)\left(x_{i}-x\right)}{\sum_{i=1}^{n}G\left(x_{i}-x/h\right)w\left(x_{i}\right)}. \end{array}$$

In formula (14), *G* represents the extended coefficient and *w* represents any constant.

Set the point set {*x*_*i*_^*∗*^}, *i*=1,2,…, *n* of the football game video image, which represents the points in the area where the football game video target is located, and the regional center point is *x*_0_. Take the regional range of the moving target as the basis to normalize the target area. Therefore, for the target template referenced by the center point *x*_0_ of the video image area, the probability distribution of *x*_*i*_ color at other positions can be assumed to be $q_{u}=\left\{{\hat{q}}_{u}\left(y\right)\right\},u=1,2,\ldots ,m$, and the distribution probability of video target color probability is expressed as

(15) $$\begin{array}{c} {\hat{q}}_{u}=C\sum_{i=1}^{n}k\left({\left\|\frac{x_{i}-x_{0}}{h}\right\|}^{2}\right)\delta \left[b\left(x_{i}\right)-u\right]. \end{array}$$

In formula (15), *δ* for the Crohneck function, *k*(*x*) is called the outline function of the kernel function, which assigns the weights of pixel points to different moving objects. A higher weight is given to moving target pixels that are close to the end point, and the kernel function can increase the overall stability of density estimation. The formula for calculating the nuclear density of a moving target is presented below (16):

(16) $$\begin{array}{c} C=\frac{1}{\sum_{i=1}^{n}k\left(\left\|x_{i}-x_{0}/h\right\|\right)},\sum_{u=1}^{m}\hat{q}u=1. \end{array}$$

In formula (16), *h* represents the range of the target area of the competition video, and the formula obtains the distribution $p_{u}=\left\{{\hat{p}}_{u}\left(y\right)\right\},u=1,2,\ldots ,m$ of the target color probability of a location *y* in the template of the candidate moving target. The distribution calculation formula of the color probability of a location in the candidate target is expressed by the following formula:

(17) $$\begin{array}{c} {\hat{p}}_{u}=C_{h}\sum_{i=1}^{n}\left({\left\|\frac{x_{i}^{*}-y}{h}\right\|}^{2}\right)\delta \left[b\left(x_{i}^{*}\right)-u\right],\\ C_{h}=\frac{1}{\sum_{i=1}^{n}k\left({\left\|x_{i}^{*}-y/h\right\|}^{2}\right)}. \end{array}$$

It is understood from formula (17) that the sampled point *x*_*i*_ of a moving target is expressed as a regularized grid, so that there is no relation between the *C*_*h*_ value and the *y* value. After calculating the range value between the kernel density value and the moving target area, the *C*_*h*_ value can also be determined.

Therefore, it can be understood that the target tracking process in the competition video is the process of comparing the similarity between the candidate templates and the target templates, and finding the best template for similarity is the best target location [19, 20]. The Bhattacharyya coefficient is calculated to obtain the similarity between the moving target template and the candidate template. The distribution of color probability, ${\hat{p}}_{u}\left(y\right)$ and ${\hat{q}}_{u}$ similarity, is represented by the following formula:

(18) $$\begin{array}{c} \rho \left[p\left(y\right),q\right]=\sum_{u=1}^{m}\sqrt{p\left(y\right){\hat{q}}_{u}}. \end{array}$$

The initial position of the video frame image in the current football match is represented by *y*_0_. Formula (18) is extended by Taylor as the following equation:

(19) $$\begin{array}{c} \rho \left[p\left(y\right),q\right]\approx \frac{1}{2}\sum_{u=1}^{m}\sqrt{p_{u}\left(y_{0}\right){\hat{q}}_{u}}+\frac{C_{h}}{2}w_{i}k\left({\left\|\frac{y-x_{i}}{h}\right\|}^{2}\right). \end{array}$$

Formula (19) shows that the size of y-value will be affected by the right side of the formula after the expansion of Taylor. Therefore, using the Taylor expansion formula in meanshift algorithm to expand the iteration of the similarity between the color probability distribution ${\hat{p}}_{u}\left(y\right)$ and ${\hat{q}}_{u}$ of the video image, the maximum density estimation of the target region probability of the video is obtained, and the maximum probability estimation is used to determine the latest position *y*_1_ of the target motion. After several iterations, *y*_1_ is the best position for the target tracking in the match video, thus completing the football match video for the detection of target and tracking.

## 5. Experimental Result

Moving target pixels that are close to the end point are given more weight, and the kernel function can improve the overall stability of density estimation.  Table 1 shows the formula for estimating the nuclear density of a moving object (16). The motion target image of football match video is shown in Figure 4.

Table 2 shows the time comparison between the methods in [1, 2] and the football video for the detection of target based on the background model is proposed in this paper.

By analyzing Table 2, it can be seen that the time for video for the detection of target in football match is 35 s for the methods mentioned in [1] and 46 s for the methods mentioned in [2]. The time for video for the detection of target in football match based on the background model proposed in this paper is 18 s, which is obviously better than the methods mentioned in [1, 2]. Therefore, the methods mentioned in this paper are more suitable for video for the detection of target in football match.  Figure 5 shows the comparison of the performance of the background model based for the detection of target method proposed in this paper with that in references [1, 2].

As shown in Figure 5, when the for the detection of target method proposed in document [1] detects the number of video frames, the overall detection effect of the experiment can reach 76 percent at first, but as the number of experimental frames increases, the detection effect deteriorates. When detecting the video image target, the overall detection effect of the for the detection of target method proposed in the document [1] is always worse, whereas the detection effect of the method mentioned in this paper is stable over 90%. The contour of the detected target is complete and the detection effect is good. The tracking times of the meanshift-based video target tracking algorithm presented in this work and those in [1, 2] are shown in Figure 6.

The target tracking technique presented in [2] grows with the growth in the number of video frames in each frame of a football match, as shown in Figure 6, and the tracking time increases gradually. The target tracking technique presented in [1] is essentially the same as that proposed in this study at the start of the experiment, but as the number of video frames rises, so does the tracking time. However, the time required to track a video target using the meanshift method suggested in this study is much less than the time required to follow a video target using the algorithms provided in [1, 2]. This demonstrates that the approach suggested in this study can enhance target tracking efficiency and is better suited to video target tracking in football matches.  Table 3 compares the number of iterations of the target tracking algorithm developed in this work to previous approaches.

Table 3 demonstrates that while monitoring a moving target in a football match video, the target tracking algorithm presented in this article uses less iterations than the classic target tracking method, indicating that the video target tracking performance discussed in this paper is better. The tracking errors of the meanshift-based video target tracking algorithm and the target tracking algorithm in the literature [1, 2] are compared in Figure 7.

By analyzing Figure 7, it can be seen that the video target tracking algorithm based on meanshift proposed in this paper can control the error of video target tracking by less than 10% as a whole. Although the error of the target tracking algorithm proposed in [1] is smaller than that in [2], the error is higher than that of the method proposed in this paper. As the number of video frames increases, the tracking error of the method proposed in [2] increases, so it is explained. The method mentioned in this paper can accurately track the video target of football match, and the tracking accuracy is high.

## 6. Conclusion

Due to the recent advancement in the field of sensors and other electronic technology, computer vision has become one of the broader and the most challenging research domain where researchers are eager to enable computerized devices to perceive things like humans. With the gradual improvement of image processing technology, the requirements for multi-for the detection of target are also gradually increasing. Football matches are a sport with a large number of viewers. Therefore, the processing of football match videos should also meet the needs of professionals and audiences. In order to improve the effect of football video detection and tracking accuracy, this paper detects and tracks the moving objects in football video, puts forward the methods of for the detection of target and tracking, and verifies the effectiveness of the methods through experiments. The experiments prove that the methods can effectively improve the effect of football video for the detection of target and tracking accuracy, which has a certain practical value.

## Figures and Tables

**Figure 1:** For the detection of target process of football stadium motion video image in background model.

**Figure 2:** Schematic diagram of mean value.

**Figure 3:** Mean slice offset diagram.

**Figure 4:** Motion target image of football match video.

**Figure 5:** Comparison of for the detection of target effects of different methods.

**Figure 6:** Comparison of target tracking time with different methods.

**Figure 7:** Comparison of target tracking errors under different methods.

**Table 1:** Experimental environment.

The environment	Data
The simulation environment	MATLAB
Runtime environment	Intel (R) Xeon (R) CPU E5-2609 v2
Memory	8G
Software environment	Windows 7
Integrated development environment	Visual Studio 2010

**Table 2:** Comparison of moving for the detection of target time with different methods.

Different methods for	Time (s)
Literature [1]	35
Literature [2]	46
In this paper, methods	18

**Table 3:** Comparison of tracking iteration times of different methods.

The evaluation index	In this paper, methods	The traditional method
Frames/frame	120	120
Iterations/times	96	210
Number of iterations per frame/time	0.8	1.75

## Data Availability

The datasets used during the present study are available from the corresponding author upon reasonable request.
